The article "Assessing the Adequacy of Hemodialysis Patients via the Graph-Based Takagi-Sugeno-Kang Fuzzy System" was published in 2021. Journal: Comput Math Methods Med.

# Assessing the Adequacy of Hemodialysis Patients via the Graph-Based Takagi-Sugeno-Kang Fuzzy System

**DOI:** 10.1155/2021/9036322

**Published:** 2021-07-27

**Authors:** Aiyan Du, Xiaofen Shi, Xiaoyi Guo, Qixiao Pei, Yijie Ding, Wei Zhou, Qun Lu, Hua Shi

**Affiliations:** ^1^Hemodialysis Center, The Affiliated Wuxi People's Hospital of Nanjing Medical University, 214000 Wuxi, China; ^2^Nursing Department, The Affiliated Wuxi People's Hospital of Nanjing Medical University, 214000 Wuxi, China; ^3^Anesthesiology Department, The Affiliated Wuxi People's Hospital of Nanjing Medical University, 214000 Wuxi, China; ^4^School of Electronic and Information Engineering, Suzhou University of Science and Technology, 215009 Suzhou, China; ^5^Yangtze Delta Region Institute, University of Electronic Science and Technology of China, 324000 Quzhou, China; ^6^Internal Medicine, The Affiliated Wuxi People's Hospital of Nanjing Medical University, 214000 Wuxi, China; ^7^School of Opto-Electronic and Communication Engineering, Xiamen University of Technology, 365001 Xiamen, China

## Abstract

Maintenance hemodialysis is the main method for the treatment of end-stage renal disease in China. The *Kt*/*V* value is the gold standard of hemodialysis adequacy. However, *Kt*/*V* requires repeated blood drawing and evaluation; it is hard to monitor dialysis adequacy frequently. In order to meet the need for repeated clinical assessments of dialysis adequacy, we want to find a noninvasive way to assess dialysis adequacy. Therefore, we collect some clinically relevant data and develop a machine learning- (ML-) based model to predict dialysis adequacy for clinical hemodialysis patients. We collect 250 patients, including gender, age, ultrafiltration (UF), predialysis body weight (preBW), postdialysis body weights (postBW), blood pressure (BP), heart rate (HR), and blood flow (BF). An efficient graph-based Takagi-Sugeno-Kang Fuzzy System (G-TSK-FS) model is proposed to predict the dialysis adequacy of hemodialysis patients. The root mean square error (RMSE) of our model is 0.1578. The proposed model can be used as a feasible method to predict dialysis adequacy, providing a new way for clinical practice. Our G-TSK-FS model could be used as a feasible method to predict dialysis adequacy, providing a new way for clinical practice.

## 1. Introduction

Maintenance hemodialysis is the main treatment for end-stage renal disease in China. Adequate hemodialysis not only prolongs survival time [1–3] but also reduces dialysis complications, improves quality of life, and reduces mortality. *Kt*/*V* is the most commonly used indicator to assess the adequacy of hemodialysis. The British Society of Nephrology and the Kidney Disease Outcome Quality Initiative (K/DOQI) recommend a minimum *Kt*/*V* of 1.2. The *Kt*/*V* value needs to measure the BUN level (before and after dialysis) and is calculated by the Daugirdas formula (*Kt*/*V*dau). This method requires repeated blood draws and evaluations, so it is difficult to frequently monitor the adequacy of dialysis. Currently, some clinical researchers used body monitor component (BCM) measurement to calculate the *Kt*/*V* value. However, the BCM technology requires special equipment, and the operation method has not yet formed a unified standard. The BCM technology cannot be widely developed. Therefore, it is especially important to find a more convenient, simple, and effective method to assess the adequacy of dialysis.

In recent years, machine learning (ML) has been widely used in the medical field and has achieved good results. For example, neural networks [4] and the support vector machine (SVM) [5, 6] were used to predict the dry weight (DW) of hemodialysis patients. In the field of bioinformatics, lots of ML technology have been well used in drug discovery [7–9], protein function [10, 11], and disease analysis [12].

ML-based predictive models can also be used to quickly estimate the adequacy of dialysis. This calculation method can provide a reference for clinical practice. Takagi-Sugeno-Kang Fuzzy Systems (TSK-FS) [13–15] are well known for good interpretability [16] and approximation accuracy [17, 18]. In this study, we developed an effective graph-based Takagi-Sugeno-Kang Fuzzy System (G-TSK-FS) model to predict the adequacy of dialysis.

## 2. Methods

### 2.1. Patients

From January 2018 to December 2020, this study collected the data of 250 patients from Wuxi People's Hospital, China. The criteria of selection are (1) patients over 18 years old, (2) patients without severe infection and heart failure within 30 days, (3) patients receiving maintenance hemodialysis for more than three months, (4) patients with no history of mental illness, and (5) patients who are informed and volunteered to participate in this study. The exclusion criteria are (1) patients who withdrew midway and (2) incomplete data.

All patients have received hemodialysis (HD) or hemodiafiltration (HDF) through the Fresenius machine. They were all dialyzed for four hours. The dialysate was fixed at 500 ml/min.  Table 1 shows the gender distribution, average age, mean predialysis body weight (preBW), average ultrafiltration level (UF) (the difference between weight before and after dialysis), average blood pressure, average heart rate, and average blood flow.

### 2.2. Blood Sampling

Each patient contains two blood samples: (1) before dialysis, a sample is collected from a vascular access vein without anticoagulant. Before collecting, we collected 10 milliliters of blood from those patients who used hemodialysis catheters as vascular access and (2) the other sample is obtained from the inlet of extracorporeal circulation before the end of dialysis. When the blood sample is taken, the blood flow rate will be slowed to 50 ml/min. At this time, the dialysate stops flowing and blood can be collected after 15 seconds.

The *Kt*/*V* is used as a “gold standard” for postdialysis, and predialysis eqU is calculated as

(1) $$\begin{array}{c} \frac{Kt}{V}=\frac{\ln\left(R-0.008\times \text{Thd}\right)+\left(4-3.5\times R\right)\times \text{Uf}}{\text{BW}}, \end{array}$$

where Uf is ultrafiltration, BW is postdialysis body weight, and Thd is the duration of the dialysis session in hours. *R* = *U*post/*U*pre.

### 2.3. Graph-Based TSK Fuzzy System

In this work, we use TSK-FS to predict the *Kt*/*V* of a hemodialysis patient. For a classic 1-order TSK fuzzy system, the fuzzy inference rules are defined as follows.

TSK fuzzy rule *R*^*k*^ is as follows.

If *x*_1_ is *A*_1_^*k*^∧*x*_2_ is *A*_2_^*k*^∧⋯∧*x*_*d*_ is *A*_*d*_^*k*^, then *f*^*k*^(**x**) = *p*_0_^*k*^ + *p*_1_^*k*^*x*_1_ + ⋯+*p*_*d*_^*k*^*x*_*d*_, *k* = 1, ⋯, *K*, where *A*_*i*_^*k*^ is a fuzzy subset of the *k*th rule for the *i*th input variable *x*_*i*_. *K* denotes the number of fuzzy rules. Each fuzzy rule is premised on the feature space **x** = [*x*_1_, *x*_2_, ⋯,*x*_*d*_]^*T*^. And TSK-FS maps the fuzzy sets to an output single dependent variable *y*^*o*^ by  *f*^*k*^(**x**). The output of the TSK-FS can be formulated as follows:

(2) $$\begin{array}{c} y^{o}=\overset{K}{\underset{k=1}{\sum }}\frac{\mu^{k}\left(x\right)}{\sum_{i=1}^{K}\mu^{i}\left(x\right)}f^{k}\left(x\right)=\overset{K}{\underset{k=1}{\sum }}{\bar{\mu }}^{k}\left(x\right)f^{k}\left(x\right), \end{array}$$

where *μ*^*k*^(**x**) and ${\bar{\mu }}^{k}\left(x\right)$ are the fuzzy membership function and normalized function via fuzzy set *A*^*k*^. And *μ*^*k*^(**x**) can be calculated by

(3) $$\begin{array}{c} \mu^{k}\left(x\right)=\overset{d}{\underset{i=1}{\prod }}\mu_{A_{i}^{k}}\left(x_{i}\right), \end{array}$$

where *μ*_*A*_*i*_^*k*^_(*x*_*i*_) is the fuzzy membership function of the *k*th rule under the *i*th input variable. In general, TSK-FS uses the Gaussian membership function:

(4) $$\begin{array}{c} \mu_{A_{i}^{k}}\left(x_{i}\right)=\exp\left(\frac{-{\left(x_{i}-c_{i}^{k}\right)}^{2}}{2\delta_{i}^{k}}\right), \end{array}$$

where *c*_*i*_^*k*^ and *δ*_*i*_^*k*^ are two parameters of the *i*th variable value of the fuzzy set *k*. Fuzzy C-means (FCM) is employed to estimate the following two parameters:

(5) $$\begin{array}{c} c_{i}^{k}=\frac{\sum_{j=1}^{N}u_{jk}x_{ji}}{\sum_{j=1}^{N}u_{jk}},\\ \delta_{i}^{k}=\frac{h\sum_{j=1}^{N}u_{jk}{\left(x_{ji}-c_{i}^{k}\right)}^{2}}{\sum_{j=1}^{N}u_{jk}}, \end{array}$$

where *u*_*jk*_ is the fuzzy membership of the *j*th sample under the *k*th fuzzy set by FCM clustering. *h* denotes the scale parameter. When the premise (if-parts) of the TSK-FS is determined, let

(6a) $$\begin{array}{c} x_{e}={\left(1,x\right)}^{T}, \end{array}$$

(6b) $$\begin{array}{c} {\bar{x}}^{k}={\bar{\mu }}^{k}\left(x\right)x_{e}, \end{array}$$

(6c) $$\begin{array}{c} x_{g}={\left({\left({\bar{x}}^{1}\right)}^{T},{\left({\bar{x}}^{2}\right)}^{T},\cdots ,{\left({\bar{x}}^{K}\right)}^{T}\right)}^{T}, \end{array}$$

(6d) $$\begin{array}{c} p^{k}={\left(p_{0}^{k},p_{2}^{k},\cdots ,p_{d}^{k}\right)}^{T}, \end{array}$$

(6e) $$\begin{array}{c} p_{g}={\left({\left(p^{1}\right)}^{T},{\left(p^{2}\right)}^{T},\cdots ,{\left(p^{K}\right)}^{T}\right)}^{T}. \end{array}$$

And equation (2) (then-parts) can be formulated as

(7) $$\begin{array}{c} y^{o}=x_{g}p_{g}. \end{array}$$

So, the problem of TSK-FS training can be regarded as solving linear regression:

(8) $$\begin{array}{c} \underset{p_{g}}{\min}\;E={\left(y-X_{g}p_{g}\right)}^{T}\left(y-X_{g}p_{g}\right), \end{array}$$

where **y** ∈ *R*^*N*×1^ and **X**_*g*_ = [**x**_*g*1_^*T*^, **x**_*g*2_^*T*^, ⋯,**x**_*gN*_^*T*^]^*T*^ ∈ *R*^*N*×*K*·(*d* + 1)^ are the true value to be approximated and the feature after fuzzy rule mapping, respectively. *N* denotes the number of training samples. *K* · (*d* + 1) is the dimension after *K* fuzzy rule mapping. To improve the generalization performance of the model, we add the Laplace regularization term to equation (8):

(9) $$\begin{array}{c} \underset{p_{g}}{\min}\;E={\left(y-X_{g}p_{g}\right)}^{T}\left(y-X_{g}p_{g}\right)+\beta Tr\left({\left(X_{g}p_{g}\right)}^{T}{LX}_{g}p_{g}\right)+\lambda p_{g}^{T}p_{g}, \end{array}$$

where *β* and *λ* are the coefficients of the two regularization terms. We derive formula (9) and get the solution

(10) $$\begin{array}{c} \frac{\partial E}{\partial p_{g}}=0-X_{g}^{T}\left(y-X_{g}p_{g}\right)+\lambda p_{g}+\beta X_{g}^{T}{LX}_{g}p_{g}=0\left(X_{g}^{T}X_{g}+\lambda I+\beta X_{g}^{T}{LX}_{g}\right)p_{g}=X_{g}^{T}y,\\ p_{g}={\left(X_{g}^{T}X_{g}+\lambda I+\beta X_{g}^{T}{LX}_{g}\right)}^{-1}X_{g}^{T}y, \end{array}$$

where **L** ∈ *R*^*N*×*N*^ is the Laplacian matrix, which can be calculated as

(11a) $$\begin{array}{c} L=D^{-1/2}\Delta D^{-1/2}, \end{array}$$

(11b) $$\begin{array}{c} \Delta =D-S, \end{array}$$

where **D** ∈ *R*^*N*×*N*^ is a diagonal matrix, *D*_*ii*_ = ∑_*j*=1_^*N*^*S*_*ij*_. Similarity matrix **S** ∈ *R*^*N*×*N*^ is built by cosine similarity of two feature vectors. We call this model as graph-based TSK-FS (G-TSK-FS), and the frame diagram of TSK-FS is shown in Figure 1. The least squares is employed to solve the optimization problem of G-TSK-FS.

## 3. Result

In this work, we test G-TSK-FS and other predictors on the dataset. Each model is evaluated with the root mean square error (RMSE) [5, 19], *R*-squared, and adjusted *R*-squared under 10-fold cross-validation (10-CV) [20, 21]. In addition, Bland-Altman analysis is also used to evaluate the agreement of two different methods (between clinical methods and predictive models).

### 3.1. Selection of Parameters for the Model

In order to make the model have the best prediction performance, we use the grid search method to get the best parameters of the model. G-TSK-FS has three parameters, including *K*, *λ*, and *β*. The range of these parameters is set as *K* ∈ {1, 2, 3, 4, 5, 6, 7, 8, 9, 10} and *λ*, *β* ∈ {2^−10^, 2^−9^, 2^−8^, 2^−7^, 2^−6^, 2^−5^, 2^−4^, 2^−3^, 2^−2^, 2^−1^, 2^0^}. First, we fix *β* = 2^0^ to search for the best *K* and *λ*. The search results are shown in Figure 2. It can be seen that the RMSE value is the minimum (0.1950) when *K* = 2 and *λ* = 2^−6^. Then, *K* and *λ* are set as 2 and 2^−6^ and *β* is set from 2^−10^ to 2^0^ with steps of 2 (in Figure 3). At last, the best RMSE is obtained under *β* = 2^−5^. In addition, the adjustable parameter of the kernel width of the Gaussian membership function is *h* = 2.

### 3.2. Comparison to Other Predictive Models

To evaluate the performance of our model, other predictive models are also tested on our dataset. They are linear regression (LR) [22, 23], support vector regression (SVR) [24], artificial neural network [25] based on the back propagation algorithm (ANN), and standard TSK-FS.  Table 2 shows the results of RMSE, *R*-squared, and adjusted *R*-squared. In general, the smaller RMSE (close to 0), the larger *R*-squared, and adjusted *R*-squared (close to 1) indicate that the model has better prediction performance. It can be seen from the table that our method (G-TSK-FS) obtains the smallest RMSE (0.1578) and the largest *R*-squared (0.7523) and adjusted *R*-squared (0.7222). In addition, G-TSK-FS has increased by 0.0181 (*R*-squared) and 0.0204 (adjusted *R*-squared) on the basis of TSK-FS. This shows that the model has better generalization performance after Laplace regularization.  Figure 4 shows the distribution of predicted values (all models) and true *Kt*/*V*. From the 150th to 160th samples, each model has severe jitter, which may be caused by the noise during the data collection process.

### 3.3. Bland-Altman Analysis

The Bland-Altman plot is a useful tool, which can evaluate the agreement between predictive methods and the clinical method.  Table 3 and Figure 5 show the results of five models via Bland-Altman analysis. In general, the lower the average difference (closer to 0) and the smaller the error acceptance range (95% confidence zone is between −1.96 SD and +1.96 SD), the better the agreement between the model and the clinical method. From the table, it can be seen that all methods have low average variance values. Among them, LR has the lowest value (−0.07312). In addition to LR and ANN, SVR (−18.1914 to 16.0155), TSK-FS (−18.1955 to 16.7179), and G-TSK-FS (−17.9686 to 16.3001) obtain the smaller range of agreement. It can be found in Figure 5 that the errors of LR and ANN for some points are very large, and the differences are greater than ±50%. For LR, ANN, SVR, TSK-FS, and G-TSK-FS, the ratios of disagreement interval are all close to 5%, which means that the prediction methods are equivalent to clinical methods. Generally, when the value is less than 5%, the prediction model can be completely equivalent to the clinical method. The results of the evaluation show that G-TSK-FS has the potential to help clinical evaluation of *Kt*/*V* with low cost.

## 4. Discussion

The kinetics of urea removal is very complicated [26], and blood is usually drawn to calculate *Kt*/*V*. What is more, strict blood collection procedures should be followed during dialysis. It is greatly affected by many factors, which will directly affect the calculation accuracy of the *Kt*/*V* value [27]. In our research, we found that adequate dialysis is related to age, gender [28], ultrafiltration [29], dry weight, dialyzer surface area, blood flow [30], DBP, SBP, and heart rate before and after dialysis. It is consistent with a previous study [31]. This indicates that these clinical features can be used to assess the ability of dialysis.

LR, ANN, and SVR are regression methods, which have been widely used in many fields. In our work, the TSK-FS method achieves better results. It is more suitable for our task. The results show that the value of *Kt*/*V* predicted by the G-TSK-FS is close to the clinical approach. G-TSK-FS obtains the smallest RMSE (0.1578) and the largest *R*-squared (0.7523) and adjusted *R*-squared (0.7222). In addition, the smaller range of agreement (−17.9686 to 16.3001) and the ratio of disagreement interval (close to 5%) show that it is a potential computational model to replace clinical methods.

Although clinical attention has been paid to the value of *Kt*/*V* in patients. Few scholars have used G-TSK-FS prediction and patients' clinical characteristics to predict patients' dialysis adequacy. In the field of precision medicine, more scholars pay attention to clinical prediction models [32–36]. Assessing the adequacy of dialysis requires repeated blood tests, which increases patient costs. In addition, the results of the adequacy test are affected by many factors, such as the quality of blood sample collection, the time of blood sample submission, and the reliability of test results. We study machine learning based on big data. Data related to the prediction model are clinical characteristics of patients. We use machine learning and other clinical data of the patient, which is convenient for clinical collection and noninvasive operation and will not increase the patient's payment, to calculate *Kt*/*V*.

## 5. Conclusions

Our method has made some progress in predicting *Kt*/*V*. However, we do not take the noise samples or the characteristics of the noise into account. In addition, the number of samples collected has not yet reached a certain scale. In future work, we will introduce other machine learning techniques such as sample filtering and feature selection [37, 38] to deal with various types of noise. At the same time, further expanding the patient sample size is also the work of the next step.

## Figures and Tables

**Figure 1:** The frame diagram of TSK-FS.

**Figure 2:** The RMSE under different *K* and *λ*.

**Figure 3:** The RMSE under different *β*.

**Figure 4:** The predicted and true values of *Kt*/*V*.

**Figure 5:** Bland-Altman plot analysis.

**Table 1:** Statistics of the studied population.

Feature	Value
Age	57.51 ± 13.582
Sex (male/female)	144/106
Urine volume (≤100 ml/>100 ml)	229/21
Dry weight (kg)	62.042 ± 12.8788
Vascular access (fistula/catheter)	209/41
Dialysis model (HD/HDF)	216/34
Dialyzer membrane area (m^2^) (1.2/1.4/1.8/2.2)	8/54/158/30
Ultrafiltration (ml)	2186.02 ± 1074.408
Systolic pressure (predialysis) (mmHg)	142.18 ± 20.941
Diastolic pressure (predialysis) (mmHg)	73.98 ± 12.907
Heart rate (predialysis)	74.82 ± 10.747
Systolic pressure (postdialysis) (mmHg)	130.7 ± 17.204
Diastolic pressure (postdialysis) (mmHg)	71.47 ± 11.094
Heart rate (postdialysis)	74.73 ± 9.676
Blood flow volume (ml/min)	274.36 ± 26.202
Conductivity (ms/cm)	14.50 ± 8.003
Venous pressure (mmHg)	123.70 ± 37.318
Transmembrane pressure (mmHg)	76.22 ± 34.528
Calcium concentration of dialysate (mmol/l) (1.25/1.5/1.75)	51/183/16
Dialysate temperature (°C) (35.5/36/36.5/37)	67/123/49/11
Predialysis weight (kg)	63.73 ± 13.593
Postdialysis weight (kg)	61.75 ± 12.91

**Table 2:** Comparison on existing methods via 10-fold cross-validation.

Method	RMSE	*R*-squared	Adjusted *R*-squared
ANN	0.2200	0.5184	0.4598
LR	0.1992	0.6051	0.5571
SVR	0.1615	0.7405	0.7089
TSK-FS	0.1634	0.7342	0.7018
G-TSK-FS	0.1578	0.7523	0.7222

**Table 3:** Bland-Altman plot analysis for different models.

Model	Average difference with true *Kt*/*V* (%)	Limits of agreement (%)		
		Lower limit	Upper limit	Number of disagreement interval
LR	−0.07312	−26.5869	26.4407	15/250
ANN	0.5469	−27.6568	28.7505	14/250
SVR	−1.0880	−18.1914	16.0155	14/250
TSK-FS	−0.7388	−18.1955	16.7179	18/250
G-TSK-FS	−0.8342	−17.9686	16.3001	15/250

## Data Availability

The data used to support the findings of this study are available from the corresponding authors upon request.
